RETRACTED

# Application of Scanning Magnetic Resonance Imaging in the Diagnosis of Prenatal Placental Implantation and Related Care

**DOI:** 10.1155/2022/4883989

**Published:** 2022-06-01

**Authors:** Qiuping Lin, Bizhu Li, Shuyun Chen, Cairu Lin, Zhixia Lin, Fengjiao Zhang, Xiaojiao Luo, Yulin Chen, Biyu Wu

**Affiliations:** ^1^Department of Obstetrics and Gynecology, The First Hospital of Quanzhou Affiliated to Fujian Medical University, Quanzhou, Fujian 362000, China; ^2^The First Hospital of Quanzhou Affiliated to Fujian Medical University, Quanzhou, Fujian 362000, China

## Abstract

In order to solve the problem of scanning magnetic resonance imaging in prenatal diagnosis, the application and research of placental implantation have been proposed. Placental implantation is a serious obstetric emergency, which refers to the abnormal attachment of placental villi caused by the dysplasia of decidual basal layer. A study from the United States showed that the incidence of placental implantation in pregnant women during delivery increased from 9.9/30000 to 11.6/20000 from 2006 to 2019, which increased the risk of prenatal or postpartum hemorrhage, hysterectomy, stillbirth, abdominal organ injury, and so on. Clinically, patients can show severe prenatal or postpartum hemorrhage, postpartum placental retention, uterine perforation, and secondary infection, which may seriously endanger the lives of pregnant mothers and fetuses. Placental implantation can also have no obvious symptoms before delivery, which leads to insufficient prenatal diagnosis. Gielchinsky retrospectively studied 410 patients with placental implantation and found that only 9 patients were detected by prenatal ultrasound or magnetic resonance imaging (MRI), and the detection rate was only 6.6%. It can be seen that if the accurate diagnosis of placental implantation can be made before prenatal or symptoms appear, clinical intervention treatment can be carried out in time to reduce the probability of hysterectomy and improve the examination means of patients' prerecovery. At present, studies at home and abroad suggest that it has good clinical application value and research prospect in the clinical diagnosis of placental implantation.

## 1. Introduction

Placental implantation is an abnormal placental implantation caused by the local deletion and interruption of the decidua fundus due to the hypoplasia or injury of the uterus, and the placental chorionic trophoblast invades the myometrium through the missing part, even breaks through the serosa, and involves the tissues and organs next to the uterus. According to the depth of placental villi implanted into the myometrium, they are divided into three types.

① Adherent placenta accreta refers to placental villi attached or adhered to the superficial muscle layer, but did not invade the deep muscle layer. ② Placenta implanta (placenta impleta) is that the placenta is implanted into the deep muscle layer without reaching the serosa layer. ③ Placenta perforta is the most serious type of placental villi penetrating the muscular layer and involving the serosa layer and even adjacent tissues and organs. The risk factors of placenta implantation are often related to endometrial trauma, endometrial dysplasia, and other factors. Because the cause of placental implantation may be endometrial damage, in addition to cesarean section, multiple uterine cleaning history, other intrauterine operation history, and intrauterine infection are also risk factors of placental implantation. Other studies have shown that older pregnancy (age > 35 years) is also one of the independent risk factors of placenta implantation. Some scholars have shown that assisted reproductive technology is another independent risk factor for placental implantation, as shown in Figure 1.

RETRACTED

## 2. Literature Review

Placental implantation is a lesion caused by hypoplasia of uterine decidua and invasion of villous tissue into uterine myometrium. Pathologically, placental implantation without decidua as an intermediary is called placental implantation. Placental implantation can be classified according to the depth of placental villi invading the myometrium, which can generally be divided into three types. Adherent placenta refers to the villi attached to the myometrium of the uterus. This type may be stripped by itself. If part of the uterine cavity remains, it can be stripped manually. Placenta accreta is due to the invasion of villi into the myometrium. At this time, it is difficult for the placenta to peel off by itself. Generally, it cannot be peeled off manually, but the overall depth has not reached the serosa layer. Penetrating implantation means that the placental villi invade the myometrium and penetrate the serosa, invade the bladder or infiltrate the parauterine tissue, and the surrounding blood flow is rich. Usually, hysterectomy and even bladder repair are needed. Once placenta implantation occurs, it is a serious obstetric complication, an important cause of postpartum hemorrhage, puerperal infection, and uterine perforation and a great threat to the life and health of pregnant women and perinatal infants. 0'Brien and others reported that the incidence rate was about 2/640 to 1/920002 in 1997. But in recent years, the incidence rate of placenta accreta has increased due to the increase of age and age of uterus and the increase of intrauterine operation [1].

RETRACTED

Prince and others believe that half-Fourier single excitation fast spin echo sequence (Haste) is the best sequence for the diagnosis of placental implantation, which is better than two-dimensional fast steady-state precession sequence (TrueFISP). The main reason is that it has fast scanning speed, reduces motion artifacts, and can obtain high-quality images [2]. Saunders and others believe that HASTE sequence signal is insensitive to fetal movement compared with TrueFISP sequence, produces less artifacts, and increases the resolution between tissues with different water content [3]. Some researchers also used single-shot fast spin echo (FSE), fast spin echo (TSE), and fast steady-state precession sequence to evaluate the placental position and the depth of invasion to the surrounding tissues. Others used T1 fat suppression sequence image to evaluate the situation of periplacental hemorrhage. Ghafoori and others did not find that diffusion weighted imaging can improve the accuracy of MRI in the diagnosis of placental implantation. Foreign scholars have found that the signal difference between placenta and uterine muscle wall of DWI sequence with *B* = 1000 s/mm^2^ is more obvious than that of T2WI [4]. In the study of postpartum placental implantation, Terpos found that in DWI sequence, high-signal placenta and relatively low-signal uterine wall were more obvious than T2WI image [5]. Venkatasubramanian et al. proposed that the local bulge of bladder and the invasion of other tissues in pelvic cavity are also strong evidence of placental implantation. Aiming at the imaging signs of uneven signal in placenta, MD proposed that it may be related to the presence of bleeding, dark zone in placenta and increased blood vessels [6]. Ireland studies believe that the appearance of intraplacental dark zone is the strongest evidence of placental implantation, followed by the discontinuity of uterine myometrium and the invasion of adjacent pelvic organs [7]. Duncan believes that placental implantation has the following specific signs. ① The lower segment of the uterus is convex or swollen. ② The placental signal is obviously uneven. Prenatal manifestations during implantation can have different audiovisual characteristics [8]. Wang and others showed that the three-dimensional color Doppler ultrasound image of placental implantation had the following characteristics. ① The blood vessels around the placenta were increased and irregular. ② Pulse perfusion or turbulence is accompanied in the dark area of echo; that is, the blood flow of placental cavity is formed [9]. Yuan and others analyzed 8 patients with lacunar blood flow sonograms by ultrasound and confirmed that 7 cases were placenta accreta, which may be related to the abnormal microvascular dynamics in the villous space. The formation of lacunar blood flow may be due to the low decidual response of such placentas, resulting in the invasion of extravillous trophoblasts into the deep muscle layer. At this time, the blood vessels originally limited to the spiral arterioles expand and then extend to the larger arcuate artery. The high pulse pressure blood flow of the deep artery forms the lacunar blood flow under ultrasound [10].

RETRACTED

Based on the current research, the application and research of placental implantation are proposed. Placenta accreta refers to the abnormal attachment of placental villi caused by the dysplasia of decidual basal layer. It is a serious obstetric emergency. In recent years, with the increase of intrauterine operation, the incidence of placental implantation is increasing year by year. Due to the differences in ethnic genetics and diagnostic level between regions, the current literature reports that the incidence of placental implantation ranges from 3/543 to 2/2205. Its complications mainly include injury of adjacent organs, intrauterine infection, and massive bleeding caused by incomplete separation of placenta during delivery. In addition, spontaneous uterine rupture in the second and third trimester of pregnancy, hemorrhagic shock, and intraperitoneal hemorrhage are also important causes of maternal death. Therefore, clinical correct and timely diagnosis of placental implantation is conducive to full prenatal preparation, reduce the complications caused by placental implantation, and then reduce the mortality of pregnant women and perinatal infants [11].

## 3. Application of Magnetic Resonance Imaging in the Diagnosis of Prenatal Placental Implantation and Related Nursing Research

### 3.1. Application of MRI in the Diagnosis of Placenta Previa and Placental Implantation

Placenta previa means that the lower edge of the placenta is close to the inner mouth of the cervix, and the distance is less than 3 cm. Placental implantation is decidual dysplasia, which leads to the invasion of placental villi into the myometrium, or serosa in severe cases, and may even involve the concave of adjacent pelvic organs. Placenta accreta is the main reason for maternal perinatal hemorrhage and postpartum hysterectomy. Placenta accreta is an important factor in incidence rate and mortality of pregnant women. The increasing prevalence of placental implantation may be related to the increasing proportion of elderly pregnant women and previous history of abortion and/or cesarean section. Accurate and timely diagnosis provides an important basis for the formulation of clinical operation plan. In the past, the imaging diagnosis of placental related diseases mostly relied on ultrasound, but there is an urgent need for an imaging that can provide more information [12].

RETRACTED

#### 3.1.1. Risk Factors of Placenta Previa and Placental Implantation

The specific etiology of placenta previa and placental implantation needs to be confirmed by further research, but a large number of studies have found that multiple intrauterine operations are high-risk factors. Cesarean section is an important risk factor. With the increase of cesarean section rate, placenta implantation incidence rate is also on the rise. The study found that the two independent risk factors of placental implantation were placenta previa and elderly pregnant women (age ≥ 36 years). Classification of placenta previa and pathological classification of placental implantation placenta previa is divided into three types according to the distance between the lower edge of placenta and the cervical opening. When the lower edge of the placenta is less than 3 cm away from the cervical opening but does not reach the cervical opening, it is called marginal placenta previa. When the lower edge of the placenta partially covers the cervical opening, it is called partial placenta previa, and when the lower edge of the placenta completely covers the cervical opening, it is called complete placenta previa. Placental implantation can be divided into three types according to the depth of villi infiltration into the myometrium: placental adhesion refers to the insertion of placental villi into the myometrium; placental implantation refers to the penetration of placental villi into the myometrium; penetrating placenta refers to the penetration of placental villous tissue into the serosa of the uterus [13].

#### 3.1.2. Clinical Manifestations of Placenta Previa and Placental Implantation

Placenta previa is easy to cause painless vaginal bleeding in the second and third trimester of pregnancy. Generally speaking, the lower the position of placenta previa, the earlier the bleeding time and the more bleeding times. It can cause potentially life-threatening serious complications, including anemia, shock, disseminated intravascular coagulation, uterine rupture, and fetal distress [14].

Placental implantation is usually characterized by prolonged third stage of labor or partial placental residue, which can cause postpartum hemorrhage and infection. Placenta accreta is a high-risk factor for uterine varus. Placenta previa and placental implantation are important causes of perinatal bleeding [15].

#### 3.1.3. Clinical Manifestations and Classification

According to the degree of placenta implantation into uterine myometrium, it can be divided into ① adherent placenta (shallow implantation), with only placental villi attached to the myometrium of the uterus; ② implantable placenta (deep implantation), the placental villi invaded the myometrium deeply; ③ penetrating placenta (deeper implantation), the placental villi invade deep into the serosa of the uterus and even penetrate the serosa to reach the bladder or rectum. In addition, according to the different degrees of placental attachment and its implantation and penetration area, it can be divided into partial placental implantation and complete placental implantation [16].

RETRACTED

There are great differences in clinical manifestations according to the depth, scope, and location of placental implantation: pregnant women with shallow placental implantation depth and small implantation range may have no special manifestations during pregnancy. During delivery and after fetal delivery, some patients may have difficulty or even no placental stripping; pregnant women with deep placental implantation and a wide range of placentas are often characterized by nonseparation of the placenta and even active massive bleeding during delivery. More serious is the rupture of the uterus in the middle and third trimester of pregnancy, resulting in massive abdominal bleeding, which endangers the lives of mothers and infants [17].

### 3.2. Differential Diagnosis of Placenta Previa and Placental Implantation

Sagittal T2-weighted image is considered to be the main sequence to judge placenta previa. It mainly measures the distance between the lower edge of the placenta and the internal orifice of the cervix. It is easier to distinguish normal placenta or placenta previa and different types of placenta previa. The correct diagnosis of placental implantation is directly related to the choice of clinical treatment strategies, so the relevant differential diagnosis is very important. (1) Differentiation between normal placenta and slight placental implantation, i.e., placental adhesion: it mainly depends on whether the signal of uterine junction zone is continuous, but sometimes it must be distinguished by some indirect signs, such as the loss of normal pear shape in the lower segment of the uterus or the low-signal dark zone of T2-weighted image in placenta. (2) Identification of placental adhesion, placental implantation, and penetrating placental implantation: some scholars believe that it is extremely difficult to identify placental adhesion and placental implantation when there is no invasion of parauterine tissue. At this time, it mainly depends on the interruption of uterine wall signal. When there is parauterine infiltration and the most common bladder invasion, it indicates penetrating placental implantation. (3) The main distinguishing point between postpartum placental detachment and postpartum placental implantation is whether the uterine junction zone is complete. When MRI plain scanning is difficult to distinguish, enhanced scanning is widely used as a better examination method. The blood supply of placenta accreta is rich, and obvious enhancement can be seen on enhanced scanning [18].

RETRACTED

### 3.3. Relationship between Placenta Previa and Placental Implantation

Placenta previa and placenta accreta are common placental-related diseases. Accurate diagnosis plays an important role in improving the prognosis. Existing studies have not fully explained the causes of placenta previa and placental implantation, but existing studies have shown that the placental implantation rate of pregnant women with placenta previa is 9%, while that of pregnant women without placenta previa is reduced to 0.006%. It can be seen that placenta previa is a high-risk factor of placental implantation. In other words, there is no necessary connection between the two, but in this study, because the enrolled patients have been confirmed as cases of placenta previa, some data can be used as a reference for the exploration and research of placenta previa with placenta implantation [19].

In recent years, it has been called dangerous placenta previa with a history of cesarean section and placenta previa. The reason is that the probability of placenta implantation in this case is greatly increased, especially placenta accreta or even penetrating placenta implantation, which will be involved in the later discussion [20].

### 3.4. High-Risk Factors of Placenta Implantation

Studies have shown that the incidence of placental implantation in recent years has increased 13 times compared with that in the early 20th century, which increases the risk of prenatal or postpartum hemorrhage, hysterectomy, stillbirth, abdominal organ injury, and so on. Clinically, patients can show severe prenatal or postpartum hemorrhage, postpartum placental retention, uterine perforation, and secondary infection, which seriously endangers the safety of pregnant mothers and fetuses.

First, the occurrence of placental implantation may be related to previous endometrial injury. Washecka and others found through 23 pregnant women diagnosed with placental implantation induced abortion, excessive curettage, multiple abortion, intrauterine infection, high number of pregnancies and births, history of placental detachment by hand, endometritis, and other history that may damage the endometrium are closely related to the occurrence of placental implantation. In this study, 46 patients in the placenta implantation group had a history of curettage, myomectomy, and cesarean section, while only 46 patients in the nonplacenta implantation group had a history of endometrial injury, which also confirmed that endometrial injury may increase the risk of placenta implantation. The possible mechanism of this process is that the endometrial basal layer is destroyed due to the above operating factors, and the endometrial functional layer cannot be effectively repaired due to various reasons. When pregnancy occurs again, the basal decidua at the implantation site may be stunted or even absent. At this time, the villi will become an implantable placenta by directly implanting into the myometrium [21].

RETRACTED

## 4. Experiment and Research

### 4.1. Comparison of Consistency between MRI Diagnosis of Placental Implantation and Surgical or Histopathological Results

In this study, method B has the highest diagnostic accuracy, so method B is compared with surgical and pathological results. Method B was used to diagnose 18 cases of PIA and 26 cases without PIA. There were 31 cases with PIA and 13 cases without PIA. The PIA diagnosis of MRI was statistically correlated with intraoperative diagnosis and histopathological diagnosis. The kappa coefficient test between them has good consistency (kappa = 0.624); that is, MRI diagnosis (method B) PIA has good consistency with surgical diagnosis and pathological diagnosis.  Table 1 shows the cross list of MRI results (method B) and surgical pathological results.

### 4.2. Analysis of MRI Signs of Placental Implantation

There were 62 abnormal MRI signs in this group, of which 10 cases showed only one abnormal MRI sign, including 7 FP cases and 3 TP cases in method A. 61 signs appeared in the PIA group, including 16 cases of interruption of uterine boundary, 7 cases of interruption of myometrial signal, 4 cases of bladder changes (0 signs of invasion of other adjacent uterine tissues), 18 cases of intraplacental dark zone, 8 cases of intraplacental blood vessels, and 9 cases of uterine dilatation. 11 abnormal signs appeared in the non-PIA group, including 3 cases of intraplacental dark zone, 6 cases of interruption of uterine boundary, 2 cases of interruption of myometrial signal, 1 case of bladder change, 1 case of intraplacental blood vessel, and 2 cases of uterine dilatation. Fisher's exact probability method was used to compare the placenta implantation group with the nonimplantation group. It was found that there were statistically significant differences between the two groups in three signs: intraplacental dark zone, focal interruption of uterine boundary, and lower uterine enlargement, as shown in Table 2 [22].

RETRACTED

### 4.3. Comparison between MRI and Ultrasound Diagnosis of Placenta Previa

In this study, 56 patients were diagnosed as placenta previa after cesarean section. The diagnostic coincidence rate of ultrasound was 79.36% (47/67), and the diagnostic coincidence rate of MRI was 99.00%. After comparison, the diagnostic coincidence rate of the two examination methods was statistically significant, that is, *P* < 0.09. In this study, 10 cases of complete placenta previa were misdiagnosed as marginal placenta previa and partial placenta previa by ultrasonography, and 1 case was missed. In contrast, there were no missed or misdiagnosed cases in MRI diagnosis, and the diagnostic coincidence rate was 99.00%. See Table 3 [23].

### 4.4. Analysis of MRI and Color Doppler Ultrasound in the Diagnosis of Placental Implantation

The pathological results (gold standard examination) of 77 patients with placental implantation (PIA) were confirmed in 28 cases and 27 patients without placental implantation. MRI showed that PIA was positive in 32 cases and negative in 24 cases; 9 cases of positive diagnosis were confirmed as normal placenta by the gold standard, and 24 cases of negative diagnosis were confirmed as normal placenta by the gold standard, so 9 cases were misdiagnosed without missed diagnosis. Color Doppler ultrasonography showed that 20 cases were PIA positive and 36 cases were negative; 4 positive cases were confirmed as normal placenta after operation, and 12 negative cases were confirmed as placenta implantation by gold standard, so 4 cases were misdiagnosed and 12 cases were missed. The coincidence rate of MRI in the diagnosis of placental implantation was 83.93%, and that of ultrasound in the diagnosis of placenta previa was 78.43% [24]. The comparison of MRI and color Doppler ultrasound diagnosis results of PIA is shown in Table 4.

### 4.5. Relationship between Diagnosis of Placental Implantation and Age Distribution of Patients

Age distribution of 104 patients with suspected placental implantation: 23 (46.1%) in the group without placental implantation and 11 (21.8%) in the group with placental implantation within the age range of 20-29; 17 (35.3%) in the group without placenta implantation and 21 (39.6%) in the group with placenta implantation within the age range of 30-34. There were 11 (22.6%) in the nonplacenta implantation group and 21 (37.6%) in the placenta implantation group. The relationship between diagnosis and age distribution of patients with placental implantation is shown in Table 5.

### 4.6. Research Object

From January 2017 to December 2018, 54 pregnant women with suspected placental implantation and prenatal MRI in Hulunbuir Hospital were selected as the research objects. The age of pregnant women was 24~41 years old, and the gestational weeks were 28~38 weeks at the time of MRI examination. In this group, 6 cases were primipara, the other 48 cases had one or more pregnancies, 26 cases had a history of cesarean section, 3 cases had a history of secondary cesarean section, and 0 cases had a history of three or more cesarean sections. 13 cases had a history of spontaneous labor. 27 cases had a history of one or more intrauterine operations such as curettage or hysteroscopy [25].

RETRACTED

#### 4.6.1. Preparations before Inspection

It is recommended that pregnant women hold their urine moderately to make the bladder in a semifilled state so that the urine can form a clear contrast with the bladder wall. It is not recommended to overfill, which will cause pregnant women unable to tolerate the examination or produce motion artifacts due to discomfort. Before the examination, eliminate the absolute contraindications and relative contraindications of MRI, remove the magnetic clothes and articles on the patient, inform the precautions, and appease the emotion so that the pregnant woman can better cooperate with the examination.

#### 4.6.2. MRI Scanning Sequence and Parameters

Scanning orientation includes horizontal position, sagittal position, and coronal position. MRI scanning sequences include coronal balanced steady-state acquisition (FIESTA), single-shot FSE (SSFSE), horizontal and sagittal balanced steady-state acquisition (FIESTA), and sagittal single-shot FSE (SS-FSE). In the fast version recovery motion inhibitory (firm) sequence, the coronal position was scanned first, the sagittal position was scanned parallel to the long axis of the placenta, and the axial position was scanned perpendicular to the long axis of the placenta. The positioning lines were copied between the sequences in the same direction.

As there are still some disputes about the safety of contrast medium to the fetus and there are no relevant technical guidelines or specifications for pregnant women to use contrast medium in China, enhanced scanning is not used as a routine examination in this study. The scanning parameters are shown in Table 6.

## 5. Conclusion

MRI provides a more accurate, objective, and comprehensive image diagnosis for the diagnosis of patients with placental-related diseases. Some scholars have proposed that MRI should be used as the routine examination P3 of placenta previa and suspected cases of placental implantation. It has broad application prospects in clinic and will better serve the majority of patients. In addition, pregnant women with intravesical hemorrhage and placental hemorrhage in the second trimester of pregnancy can also be caused by maternal shock and placental hemorrhage, which can also be harmful to pregnant women. MRI has become an important method for the diagnosis of placenta previa and placental implantation because of its high soft tissue resolution and large imaging range. The application of MRI can improve the accuracy of placenta implantation diagnosis. Through the continuous exploration of the image characteristics of MRI placental-related diseases, MRI will play an increasingly important role in the diagnosis of placenta previa and placental implantation, providing a broader space for clinical work.

RETRACTED

## Figures and Tables

**Figure 1:** MRI diagnosis of placental implantation.

**Table 1:** Surgical diagnosis and pathological diagnosis.

Adhesiveness		Implantation	Pierce through	No PA	Total
Adhesiveness	12	5	7	2	0
Implantability	11	5	4	10	20
Penetrability	0	5	4	2	12
Total	23	15	15	14	22

**Table 2:** Comparative analysis of MRI abnormal signs in the PA group and the non-PA group.

Abnormal MRI findings	PIA group	Non-PIA group	*X* ^2^	*P* value
Intraplacental vessels	20	3	11.36	0.003
Uterine enlargement	16	1	2.36	0.062
Interruption of uterine boundary	14	5	3.23	0.23

**Table 3:** Comparison of MRI and ultrasound diagnosis of placenta previa.

MRI examination	Ultrasonic examination		
Consistent with postoperative diagnosis	46	12	58
Does not meet the postoperative diagnosis	1	2	1
Total	47	14	59

**Table 4:** Comparison of MRI and color Doppler ultrasonography in diagnosis of placenta previa.

MRI examination	Color Doppler ultrasound examination		
Postoperative diagnosis of color Doppler ultrasound	12	16	7
Color Doppler ultrasound does not meet the postoperative diagnosis	3	3	1
Total	15	19	8

**Table 5:** Relationship between diagnosis and age distribution of patients with placental implantation.

Age	Placenta-free group	Placenta implantation group
30-39	24	15
40-49	15	23
>30	13	26

**Table 6:** MRI scanning parameters.

	SS-FS	FRIM	ERTA
Repetition time	Infinity	4.0	7
Layer thickness	80	1.9	4.9
Echo time	6	9	2
Number of layers	20-40	30-40	50

## Data Availability

The data used to support the findings of this study are available from the corresponding author upon request.
